# Dose selection of central or peripheral administration of sufentanil affect opioid induced cough?: a prospective, randomized, controlled trial

**DOI:** 10.1186/s12871-018-0502-z

**Published:** 2018-04-10

**Authors:** Jiabei He, Ling Zhu, Huichen Zhu, Xinyu Gu, Peiying Li, Yuting Yang, Liqun Yang

**Affiliations:** Department of Anesthesiology, Renji Hospital, School of Medicine, Shanghai Jiaotong University, Shanghai, 200127 China

**Keywords:** Sufentanil, Cough, Peripheral, Central

## Abstract

**Background:**

Opioid-induced cough (OIC) is one of the most common complications of opioids during anesthesia induction. This study was designed to assess the incidence of OIC mediated by different intravenous route.

**Methods:**

A total of 102(ASA I-II) scheduled for elective surgery under general anesthesia were randomly allocated into two groups: central vein group (group CV, *n* = 51) and peripheral vein group (group PV, n = 51). The incidence, onset time and severity of OIC were evaluated within 1 min just after sufentanil injection during induction. Meanwhile, heart rate (HR) and blood pressure (BP) were also recorded to assess the hemodynamic changes.

**Results:**

The incidence of OIC was 10/51 (20.4%) in group CV and 16/51 (32%) in group PV, patients received central venous administration of sufentanil experienced less OIC compared with those injected by peripheral venous route (*P* < 0.05), as well as a significantly lower incidence of severe OIC (P < 0.05). Nevertheless, the onset of OIC and hemodynamic data were comparable between two groups (*P* > 0.05).

**Conclusion:**

Our study indicates that sufentanil administration by central venous route reduces the incidence and severity of OIC, but without significant changes in hemodynamic status.

**Trial registration:**

Chinese Clinical Trial Registry with registration number ChiCTR-IOR-15006075. Registered 28 February 2015.

## Background

Opioid are frequently used as a pre-induction adjunct because of their strong analgesic properties, relatively short duration of action and minor disturbance of cardiovascular stability. Opioid-induced cough(OIC) during induction of general anesthesia is a common complication of opioids, with a reported incidence varying between 2.7 and 65% [1, 2]. Even though OIC appears to be transient and harmless in most cases, this pathological condition may specially result in life-threatening consequences in patients for example with a compromised central nervous system (CNS), open eye injury, and cardiovascular diseases [3] which require an absolutely stable hemodynamic status and intracranial or intraocular pressure during anesthesia induction. Various clinical interventions have been reported to reduce OIC, including pretreatment with lidocaine [4], propofol [5], magnesium [6], or steroids [7] and with non-pharmacological intervention such as opioid dilution and slow injection [8]. However, there is limited information about whether administration route can influence OIC incidence.

Sufentanil is a potent opioid and stands out from other opioids because of its fast onset and strength of analgesic action, which also makes it as an ideal option and one of the most used opioids in anesthesia induction. However, sufentanil was identified to bring on OIC even with small doses [9]. Therefore, interventions to reduce sufentanil-induced cough do have clinical significance.

In this prospective, randomized, and controlled study, we investigated whether administration route of sufentanil can change the incidence of OIC.

## Methods

This study was approved by the institutional ethics committee (IRB of Renji Hospital, School of Medicine Shanghai Jiaotong University) and registered at Chinese Clinical Trial Registry with registration number ChiCTR-IOR-15006075. This manuscript adheres to the applicable Equator guidelines.

The study was conducted between April 2015 and March 2016. A total of 102 patients, aged 18–65 years, classified as American Society of Anesthesiologists (ASA) physical status I-II, and scheduled for elective surgery under general anesthesia were enrolled in this study. The exclusion criteria included a history of asthma or chronic obstructive pulmonary disease (COPD), upper respiratory tract infection in the last two weeks, smoking, bronchodilator or steroid therapy, chronic administration of opioids, anti cough medication or angiotensin-converting enzyme(ACE) inhibitors. Patients diagnosed to have increased intracranial or intraocular pressure were also excluded. They were randomly assigned to central venous (group CV) and peripheral venous group (group PV) using computer-generated random numbers by Microsoft® Excel 2003. Every randomization code was prepared in an envelope by a nurse who was no longer engaged in the following steps. Neither were other medical staff who did data collection and anesthesia induction.

No premedication was administered before surgery. Upon arrival in the operating room, monitoring was accomplished by heart rate, invasive arterial blood pressure, respiratory rate and oxygen saturation (S/5 Anesthesia Monitor; Datex-Ohmeda, Madison, WI, USA). Patients in Group CV received a F16 single lumen central venous catheter (Arrow®, Arrow International Inc., Reading, PA, USA) inserted via the right jugular vein after local infiltration of 1 ml lidocaine, while a 18-gauge cannula was also inserted into the forearm or dorsum of the hand and connected to a three-way stopcock among patients in Group PV. Intravenous perfusion was maintained with ringer’s lactate at the rate of 6 ml.kg^− 1^.h^− 1^ after venous catheterization finished.

Anesthesia induction was initiated with a 0.05 mg/kg of midazolam, which was followed by a 0.35 μg/kg of sufentanil, that was injected and finished within two seconds. The incidence, occurrence time and severity of cough in patients were evaluated by a nurse within 1 min after the injection of sufentanil. The occurrence of cough as ‘yes’ or ‘no’, within a 1-min period, and the onset time of cough (from the start of the infusion to the beginning of coughing) were recorded immediately after injection. Depending on the number of coughs observed, the cough severity was graded as mild [1, 2], moderate [3–5] and severe (>5). Systolic and diastolic blood pressure (SBP and DBP, respectively) and HR were recorded before the injection of sufentanil (T_0_) and 1 min after the injection of sufentanil (T_1_). Anesthesia induction was finished with subsequent propofol 2 mg/kg and 0.9 mg/kg of rocuronium, which was followed by an orotracheal intubation. Anesthesia was maintained by 1–2 Mac of sevoflurane with 40% of O_2_ and 60% of air. Opioids and neuromuscular blocking drugs were administered according to the standard anesthetic protocol. All the patients were transferred to PACU and monitored for at least 1 h after surgery.

Our sample body was determined based on a pilot study: we took our primary end point as the detection of 30% reduction in of the incidence of sufentanil-induced cough in PV group, and to have a study power of 90% with a one-sided test and 0.05 significance. A total of 42 patients per group would be required. We have decided to enroll 54 patients in each group by considering the inevitable dropout. Data were expressed as mean ± SD, number or percentage, statistical analysis was performed with a personal computer statistical software package (Prism version 5.0; Graph-Pad Software, San Diego, CA) using independent t-test and Chi-Square test. *P* < 0.05 was considered as statistically significant.

## Results

A total of 108 patients were initially enrolled in this study, but 6 patients were dropped out because of failure in data collection and patient’s concealment of smoking history. Other 102 patients were randomly allocated into two groups as shown in Fig. 1. There was no statistical difference in demographic data in terms of age, sex, weight, height, BMI and ASA classifications. Neither was the hemodynamic changes between two groups (P>0.05, Table 1). The incidence of cough was 10/51 (20.4%) in group CV and 16/51 (32%) in group PV (Table 2), which presented a statistically significant difference (*P* < 0.05). Furthermore, patients in group CV experience significantly less frequent severe cough (1/51, 1.96%) when compared with group PV (6/51, 11.76%) (P < 0.05) (Table 2). There was no significant difference in the onset time of cough between two groups (shown in Table 2).

**Fig. 1:** Consort diagram: flow of patients through the study

**Table 1:** Demographic profiles and hemodynamic data between 2 groups

	Group CV (*n* = 51)	Group PV (*n* = 51)	*P* value
Age (years)	50.0 ± 11.1	52.8 ± 9.7	0.18
Height(cm)	165.0 ± 7.5	164.9 ± 8.6	0.94
Weight (kg)	63.2 ± 9.4	64.3 ± 10.2	0.55
BMI	23.1 ± 2.4	23.6 ± 3.0	0.36
ASA (I/II)	38/13	35/16	0.66
Sex (M/F)	28/23	28/23	1.00
SBP _T0_	143.51 ± 12.7	144.2 ± 16.2	0.81
DBP _T0_	77.2 ± 7.3	76.7 ± 8.3	0.72
HR _T0_	75.8 ± 9.9	77.2 ± 13.1	0.54
SBP _T1_	125.3 ± 16.1	125.1 ± 16.6	0.93
DBP _T1_	69.1 ± 8.5	69.3 ± 9.0	0.89
HR _T1_	76.3 ± 11.0	77.9 ± 13.2	0.50

*Group CV* central venous group, *Group PV* peripheral venous group, *SBP* systolic blood pressure, *DBP* diastolic blood pressure, *HR* heart rate, *T*_*0*_ time before injection of sufentanil, *T*_*1*_ 1 min after injection of sufentanil

Data represented mean ± SD or numbers. Independent t-test was used. A *p* value of < 0.05 was considered statistically significant

**Table 2:** Incidence and severity characteristics of sufentanil induced coughs

	Group CV (*n* = 51)	Group PV (*n* = 51)	P value
Occurrence of cough, n (%)	10 (20.4)	16 (32)	0.04^*^
Mild	4 (7.84)	5 (9.80)	0.36
Moderate	5 (9.80)	5 (9.80)	1.00
Severe	1 (1.96)	6 (11.76)	0.03^*^
Onset time of cough (s)	18.3 ± 3.0	18.5 ± 2.8	0.93

*Group CV*central venous group, *Group PV* peripheral venous group

Values are mean ± SD or numbers (percentage). Chi-Square test was used. A p value of < 0.05 was considered statistically significant

*p <0.05, group CV vs. group PV

## Discussion

Our study identified that the frequency of sufentanil-induced cough was significantly lower in patients by central venous administration route than those through peripheral route during general anesthesia induction, and the incidence of severe cough was also significantly lower among patients using central venous administration route.

Arm-to-head time was defined as the interval between the start of the injection of an echo-contrast agent into the antecubital vein and the beginning of signal amplification in the carotid artery, and was reported to be 14.3 (3.0) s (9.0–22.0 s) by Hoffmann et al. [10]. However, Blumgart and Weiss [11] detected an active deposit of radium in the right ventricle following 2.5–14.0 s after antecubital vein injection (arm-to-heart time) and estimated the pulmonary circulation time to be 5.5–17.5 s. Therefore, it was unlikely that sufentanil could enter CNS within 5 s and induce cough via CNS-located receptors, instead, the more possible explanation should be that it triggered cough by activating receptors located in the periphery, for example thorax or lung. This was supported by the study from Karlsson et al. [12], they demonstrated that the activation of μ or κ opioid receptors located in tracheobronchial tree inhibits cough and bronchoconstriction reflex. According to their presumption, a central venous administration route should be associated with a higher prevalence of OIC since it dramatically increases opioid concentration in a very short period of time. Nevertheless, it is inconsistent to our study.

The occurrence of OIC is not completely determined by local effective-site concentration. Kim JY et al. [5] suggested that the discrepancy between plasma concentration and effective-site concentration influence the occurrence of OIC as well, and the bigger the discrepancy is, the higher incidence of coughing occurs. Our study was aligned with this hypothesis: central venous route was associated with a faster increase in pulmonary drug concentration and a smaller difference between plasma and local opioid concentration. Thus, it’s reasonable that lower incidence of cough was observed in central venous route group.

Another contributor to OIC besides opioid itself is citric acid. In clinical practice, sufentanil reagents are prepared in a form of citrate salts. Notably, citric acid can initiate the cough reflex by stimulating C-fibres in the airway [13], which thereafter releases sensory neuropeptides, and causes neurogenetic inflammation and indirectly activates rapidly adapting receptors(RARs) to initiate cough. After administration of opioids through peripheral vein, citric acid can stimulate terminals of peripheral primary sensory neurons to release tachykinins substance P (SP) and neurokinin A(NKA), which further activates NK(1) and NK(2) receptors, and consequently leads to neurogenic inflammation [14], which might be another explanation of a higher incidence of OIC by peripheral administration.

Studies aimed to reduce OIC can be roughly divided into pharmacological and non-pharmacological ways. Dezocine [15], magnesium sulfate [6] and dexmedetomidine [16] have been reported to be effective to reduce sufentanil-induced cough while undesirable side-effects [17] and higher financial cost should also be considered. Non-pharmacological interventions include slow injection [18] and dilution [8]. Slow injection and dilution can lead to a reduced peak plasma concentration and that is probably the reason why OIC was suppressed. Nevertheless, slow injection may not always be practical, especially in case of emergency. In comparison with methods mentioned above, our method was safe and effective, time and cost saving.

However, there are also some limitations in our study: Firstly, the average age of the patients enrolled in this study was around 50, and age was believed to be an important confounding factor in OIC occurrence. Younger patients, especially children and infants were more vulnerable to OIC [19]. Secondly, CV administration route did not completely prevent OIC. Therefore, a combination of various effective interventions might give us a more satisfying outcome and offer a better protection against OIC. Finally, anesthesia induction was achieved by a combination of several reagents and whether the change of administration route of other drugs affect OIC was unknown and warrants to be further investigated.

## Conclusions

Our results suggested that sufentanil administered through central vein reduces the occurrence and severity of sufentanil-induced irritating cough without causing significant changes in hemodynamic status during general anesthesia induction. Therefore, central venous route could be preferred for anesthesia induction when it was applicable.
